# Explore the Link between the Improvement of Metabolic Indicators in Diabetic Rats with Sleeve Gastrectomy and Changes in the Composition of Intestinal Flora

**DOI:** 10.1155/2022/7027777

**Published:** 2022-02-18

**Authors:** Jingjing Zhang, Tao Li, Gang Yao, Apaer Shadiker, Shensen Gu, Xinling Cao

**Affiliations:** ^1^State Key Laboratory of Pathogenesis, Prevention and Treatment of High Incidence Diseases in Central Asia, Department of Nephrology, The First Affiliated Hospital of Xinjiang Medical University, Urumqi 830011, China; ^2^State Key Laboratory of Pathogenesis, Prevention and Treatment of High Incidence Diseases in Central Asia, Department of Liver Transplantation & Laparoscopic Surgery, The First Affiliated Hospital of Xinjiang Medical University, Urumqi 830011, China

## Abstract

Diabetes mellitus (DM) has become a major medical and health problem in my country and even the world. Doctors and patients have gradually realized that a new type of metabolic surgery is a way to treat diabetes. The operation is relatively simple, and the effect of the operation is no less than that of the gastric shunt. The initial hypothesis could not fully explain the blood pressure and blood sugar reduction mechanism in waist and abdominal surgery. According to requirements, they were divided into the sleeve gastrectomy group (SG group, *n* = 10) and sham operation group (SS group, *n* = 10), and corresponding measures were taken. Observe their weight changes; perform an oral glucose tolerance test (GB) before surgery and at 2, 8, and 16 weeks after surgery to evaluate the effect of surgery on improving the glucose metabolism. The postoperative GLP-1 specificity curve was detected in the two groups of patients; the immunohistochemical method was used to detect the postoperative changes of the digestive tract l cells in the two groups; RT-PCR was used to detect the mRNA transcription level of the digestive tract GLP-1 receptor. The bodyweight was significantly different 4 weeks after the operation. Food intake and bodyweight were not significantly different between the SG and SS groups. FBG: one week after operation, the SG group was significantly smaller than the SS group. The SS group was significantly lower than the SG group at 12 weeks after operation, and the SS group was significantly lower than the SG group at 14 weeks after operation. The transcription levels of c-kit mRNA and SCF mRNA in jejunum and ileum tissues are significantly different: the transcription levels of c-kit mRNA and SCF mRNA in the SG group are higher than those in the SS group, jejunum and ileum in the SG group. The number of cell 1 was significantly greater than that of the SS group. Sleeve gastrectomy can improve the regulation of the glucose metabolism in diabetic rats. The increase in small bowel motility may be related to the increase in ICC cells, intestinal cells, and GLP after gastric sleeve resection. The increase is in -1R and faster insoluble CHM in bowel motility. It has better contact with cell 1 and GLP-1R and stimulates cell 1 to secrete GLP-1.

## 1. Introduction

At present, sleeve gastrectomy is the most effective treatment of type 2 diabetes. The recovery rate of postoperative diabetes exceeds 80%, but the principle of reducing sleeve gastrectomy of type 2 diabetes is not clear, which will inevitably affect the intestinal tract [1]. Environmental and microscopy have disrupted the ecological balance of the gut with ongoing scientific studies of gut microbiota and gut glucose metabolism, and therefore, the study has become an important study by papering the changes in the gut microbiota after gastric bypass surgery [2]. The procedure was simple; below and most of the stomach, the anatomical relationship was not disrupted and the digestive system was retained. Injury continuity was minimal and had a low incidence of surgery-related complications. It is increasingly important to provide more information and clues about the potential link between gut flora and alleviating the glucose metabolism after surgery [3]. Experienced surface distribution of intestinal flora and monocyte necrosis factor CCR2, CX3CR1, intracellular monocyte necrosis factor (TNF-), interleukin 6 (IL-6), and substrate monocyte transformation; and LPS TLR4 receptor expression was found in diabetic patients. Cell surface changes in the monocyte subspecies [4]. Type 2 diabetes cannot control weight or blood sugar for a long time and cannot avoid the occurrence and aggravation of various diabetes complications. Surgery is currently the only long-term effective means for the treatment of pathological sleeve gastrectomy. Studies have shown that sleeve gastrectomy can control blood glucose while with weight loss and improve blood glucose levels in type 2 diabetes. It is caused by stimulating monocytes to slow low levels of chronic inflammation and eliminate intestinal development and effects of intestinal flora and the glucose metabolism, vertical bending of the stomach into a small cyst, about 150 cc in the stomach; when LPS enters, the increased internal circulation has shown that sleeve gastrectomy is effective in weight loss and reducing complications associated with sleeve gastrectomy [5]. Therefore, in order to further explore the specific clinical application of sleeve gastrectomy and provide a safer and effective treatment for diabetic patients, this study established a mouse model to paper and explore sleeve gastrectomy, which will be reported as follows.

## 2. Data and Methods

Three-week-old SPF SPK male rats were prepared (38.22. ± 3.24), g.SCXK (E): 2015-0003-0001365. Group and intervention: 35 sleeve gastrectomy rats were randomly divided into two different groups: the sleeve gastrectomy group (SG, *n* = 20) underwent a sleeve gastrectomy and the general group (SS, *n* = 15) underwent general surgery. After the intervention, both groups were fed regularly for 4 weeks, and then, the paper indicators were measured. Methods of gastrointestinal resection and general surgery as well as perioperative treatments are referred to existing methods. In this study, the methods of feeding and weighing significant rats and the specific operation of each index detection are described as follows.

The SS and SG groups were fed feed oil containing 20% fat (17% sardines and 3% corn) with calories of 4.85 calories of food and water. After 16 weeks of feeding, successful intraperitoneal injection of 25 mg/kg (50 mg/kg) was performed once, maintaining the original diet with free food and water after injection [6]. After 72 hours, blood was collected from the tail vein, and fasting glucose was measured using a glucose meter. 13.5 mmol/L above is the successful model. Mice were weighed for the first three days in the first week after unified surgery and then called once weekly for eight consecutive weeks. Seven additional rats were fed normally [7].

After half an hour, the amount of food was measured and the chimney residue in the stomach after half an hour and recorded its quality (g), accurate to 0.1 g.2 [8]. Feed removal method: measure the entire length of the small intestine (villus to ileum) and the transition distance from the end of the pylorus to the ileum and record the length (cm) with a precision of 0.1 cm.

(1) After disinfecting the curtain, take the midline of the upper abdominal incision downward along the sword protrusion [9]. After the rat skin was cut, the white line was exposed [10]. (2) After entering the abdomen, the abdomen is checked using a sterile cotton swab dipped in normal saline to determine the location of each organ [11]. First, the blunt raw tissue around the abdomen (spleen and stomach ligaments and liver and abdominal stents) was separated and then ligated and blood vessels cut off (5–0 mousse) [12]. Pay attention to mild exercise during release and avoid pulling hard to avoid damage to the spleen and liver [13]. (3) Check the location of the heart and pylorus, fully release the heart and eyes of the abdomen, and continue to release the mesentery on the curved side of the abdomen, approximately 5 ml from the pylorus [14]. During this period, larger vessels were connected with 5–0 mousse and then cut off with a coagulation knife to stop bleeding. Once the glomerular mesentery was confirmed without active bleeding, the free mesum was returned to the abdominal cavity [15]. (4) Cut the appetite along the length of the abdomen with small scissors and clean the abdominal contents with a wet cotton swab (the main body should be rat hair) [16]. The vessel clamp was released during the suture to avoid ischemia and swelling in the abdominal wall and to promote postoperative healing. After the suture was completed, the venous stent was removed and the blood flow to the rest of the gastric wall tissue was carefully monitored and noted for blood leakage or fluid leakage in the stump. After confirming that there were no abnormalities, the remaining abdomen was disinfected and returned in situ to the abdominal cavity [17]. After careful examination, the abdominal wall was stratified with continuous suture after disinfection. Finally, the incision skin was disinfected with Ann iodine, and the surgery was terminated [18].

Paraffin section dewaxed to water. Incubate at 3%H_2_O_2_ for 5–10 min to eliminate endogenous peroxidase activity. Rinse with distilled water and immerse in PBS x2 for 5 min (if antigen repair is required, it can be performed after this step); 5–10% normal goat serum (diluted with PBS) was sealed and incubated at room temperature for 10 min [19]. The serum was poured out without washing [20]. Add primary antibody working solution and incubate at 37°C for 1-2 hours or overnight at 4°C. Wash with PBS, x3 times 5 min. Appropriate amount of biotin-labeled secondary antibody working solution was added and incubated at 37°C for 10–30 minutes [21]. Wash with PBS, x3 times 5 min. Add appropriate amount of horseradish enzyme or alkaline phosphatase labeled streptomycin working solution and incubate at 37°C for 10–30 minutes [22]. Wash with PBS, x3 times 5 min, chromogenic agent for 3–15 minutes (DAB or NBT/BCIP), rinse, dye, dehydrate, transparent, and seal with tap water.

Total RNA was extracted from mice. Synthesis of first strand cDNA: refer to the instructions of the first-strand cDNA kit. Total RNA 1–5 *μ*g was added to a 0.5 mL microcentrifuge tube, and DEPC H_2_O was supplemented to make the total volume up to 11 *μ*L. Add 10 *μ*M oligo (dT) 12–18 1 *μ*L to the tube, mix gently, and centrifuge [23]. After heating at 70°C for 10 min, insert the microcentrifuge tube into the ice bath for at least 1 min. Add the following reagents to the mixture: 10 × PCR buffer 2 *μ*L, 25 mM MgCl 22 *μ*L, 10 mM dNTP mix 1 *μ*L, 0.1 m DTT 2 *μ*l, gently mix, centrifuge, incubate at 42°C for 2–5 min, add superscript 1 *μ*L, and incubate in the waterbath at 42°C for 50 min [24]. The reaction was terminated by heating at 70°C for 15 min. The tubes were inserted into ice, 1 *μ*l RNase *H* was added, and incubated at 37°C for 20 min to degrade the residual RNA. Store at −20°C for later use. Take the 0.5 mL PCR tube, add the following reagents successively: first strand cDNA 2 *μ*L, upstream primer (10 pM) 2 *μ*L, downstream primer (10 pM) 2 *μ*L, dNTP(2 mM) 4 *μ*L, 10 × PCR buffer 5 *μ*L, and Taq enzyme (2U/*μ*L) 1 *μ*L. Add appropriate amount of ddH_2_O to make the total volume up to 50 *μ*L. Gently mix, centrifuge, and set up PCR program. 28–32 cycles were amplified at appropriate temperature parameters. In order to ensure the reliability and accuracy of experimental results, a pair of specific primers for internal reference (such as G3PD) can be added during PCR amplification of target genes, and the reference DNA can be amplified at the same time as the control. Electrophoresis identification: agarose gel electrophoresis and UV lamp observation results. Density scanning and result analysis: the gel image analysis system was used to carry out density scanning of electrophoresis bands.

The weight changes of the two groups were compared before and after operation. Glucose was taken orally before and after surgery to observe the specific effect of the operation on improving the glucose metabolism. Postoperative GLP-1 profile of the two groups of mice was compared. The immunohistochemical method was used to detect the changes of digestive tract cells in the two groups after operation. The mRNA transcription levels of the GLP-1 receptor in digestive tract of the two groups were detected and compared.

In this study, SPSS 22.0 was used for analysis. Measurement data are expressed as mean ± standard deviation ($\bar{x}$ *±* *s*), using the *t*-test; counting data are expressed as (*n* (%)), using the c2 test, with *P* < 0.05 meaning that the difference is statistically significant.

## 3. Results and Discussion

Rat' bodyweight and feeding comparisons are given in Table 1. The results showed that there was no significant difference in bodyweight between the two groups before surgery, and the weight gain of the SG group was significantly lower than that of the SS group after surgery (*P* < 0.05). Table 1 provides rat' bodyweight and feeding.

Insulin changes in the two groups are given in Table 2. The results showed that the insulin level in the SS group was higher than that in the SG group at all time periods (*P* < 0.05).

Insulin and blood glucose changes are given in Table 3.

Bodyweight change in rats, as given in Table 4. The results showed that the weight of rats in the SG group decreased after operation, while that in the SS group increased (*P* < 0.05).  Figure 1 shows bodyweight change in rats in each group.

Internecinal transmission was observed for half an hour in the two groups, as shown in Figure 2.

## 4. Conclusion

The proportion of bacteria decreased in sleeve gastrectomy and increased in sleeve gastrectomy. Existing studies have shown that antibiotic use affects the structure of the human gut flora, but the changes caused by this effect will return to the state before antibiotic use 30 days after antibiotic cessation. Furthermore, in animal studies, changes in key metabolic indicators (e. g., bodyweight and blood glucose) after performing sleeve gastrectomy reached the lowest levels in the experimental animals at 2.4 weeks after the experiment, indicating the strongest metabolic level. The healing effect is the strongest. Considering these two factors, we decided to paper the effect of cochlear gastrectomy at 1 month after surgery on the intestinal microbiota and metabolism. The current study shows that SPS is closely associated with sleeve gastrectomy. Certain *Firmicutes* bacteria have the ability to produce H2. These bacteria can ferment plant polysaccharides in food into SCFA while producing H2. These SCFAs provide additional energy to the body. Hard is indeed found in individuals with sleeve gastrectomy. This suggests that this mechanism of the gut flora plays a key role in sleeve gastrectomy. Our study also found that the proportion of hard hair decreased after removal after weight loss, indicating that rat weight loss after surgery is not only for the reduction in food intake but also for intestinal bacteria, and the intestine is the organ where the body directly communicates with the organs. The gut is resistant to harmful components of the gut, such as the gut flora and its produced endotoxins, that enter the body's blood through the intestinal mucosa. The structure and function of this total gut is called the “intestinal barrier.” An increase in TNF-phosphomyosin shrinks the IEC backbone and cuts off connections. Claudin-1, claudin-3, occludin, and claudin-1 have also been found in the intestinal mucosa of connexin 1 and other adipose animals, and mechanical intestinal inhibition is a very important pathogen in the pathogenesis of metabolic endotoxemia.

At the same time, previous studies have found that sleeve-like surgery could promote the regeneration and release of GLP-2 and increase the levels of GLP-2. Intestinal L cells secrete peptides and intestinal epithelial-specific growth factors to promote the growth of functional intestinal mucosa, which is more important than other epithelial growth factors, where it is necessary to repair the damaged intestinal epithelium. Epithelial expression is strongly associated with proteins, thereby increasing the inhibitory effect on intestinal mucosal function. Therefore, to determine differences in intestinal permeability, we examined here whether intestinal permeability varied after GLP-2 surgery to promote exogenous GLP-2 and reduce the damage of intestinal tight junction proteins. After continuing the high-fat diet, the rectal permeability of SG decreased, followed by surgery, but SG continued to decrease after surgery. It has a great effect on the glucose metabolism and intestinal flora after passing through sleeve gastrectomy. This result is consistent with SS surgery and can provide longer glycemic lowering effects. Improving and decreased insulin sensitivity after SG surgery may be associated with intestinal permeability and chronic inflammation. In addition, although some achievements have been made in this study, there are still shortcomings. There are still some differences between rats and human bodies. Therefore, the results and mechanisms of this study need to be confirmed by further experiments in humans.

In conclusion, sleeve gastrectomy can significantly enhance the glucose metabolism, promote gastrointestinal peristalsis, and stimulate glP-1 secretion in rats, which has a good clinical application value.

## Figures and Tables

**Figure 1:** Bodyweight change in rats in each group.

**Figure 2:** Transmission ratio comparison.

**Table 1:** Rat bodyweight and feeding.

Group	Example number	Average daily food intake/g			Weight/g	
		Preoperative	Postoperative	Preoperative	After surgery, 8 weeks	The average postoperative daily weight gain was observed

SG group		33.6 ± 3.2	18.6 ± 2.2	464.6 ± 2.9	412.9 ± 2.9	0.98 ± 0.32
SS group		37.2 ± 3.6	35.6 ± 1.5	468.6 ± 3.1	493.3 ± 3.2	1.21 ± 0.22

**Table 2:** Insulin changes in rats.

Group	Preoperative				Postoperative			
	0 min	30 min	60 min	120 min	0 min	30 min	60 min	120 min

SG group	18.6 ± 2.2	464.6 ± 2.9	412.9 ± 2.9	0.98 ± 0.32	18.6 ± 2.2	464.6 ± 2.9	412.9 ± 2.9	0.98 ± 0.32
SS group	35.6 ± 1.5	468.6 ± 3.1	493.3 ± 3.2	1.21 ± 0.22	35.6 ± 1.5	468.6 ± 3.1	493.3 ± 3.2	1.21 ± 0.22

**Table 3:** Blood glucose changes.

Group	Blood glucose before surgery	After glycemic surgery
	(ng/mL)	(ng/mL)

SG group	207.6 ± 2.34	128.89 ± 4.31
SS group	83.6 ± 1.19	76.24 ± 2.45

**Table 4:** Bodyweight changes in rats.

Bodyweight (g) time	SG group	SS group	*P*

Before surgery	362.8 ± 9.3	361.5 ± 25.0	≤0.001
January after surgery	332.2 ± 34.6	379.2 ± 11.6	≤0.001

## Data Availability

The data used to support the findings of this study are available from the corresponding author upon request.
